The article "Effects of Continuous Infusion of Lidocaine under Ultrasound-Guided Cervical Sympathetic Ganglion Catheterization on Cerebral Hemodynamics and Thermal Imaging Characteristics of Head and Neck in Patients with Angioneurotic Headache" was retracted in 2023. Reasons: suspected computer-generated content; unreliable results or conclusions; concerns about the data; concerns about the results or conclusions.

# Effects of Continuous Infusion of Lidocaine under Ultrasound-Guided Cervical Sympathetic Ganglion Catheterization on Cerebral Hemodynamics and Thermal Imaging Characteristics of Head and Neck in Patients with Angioneurotic Headache

**DOI:** 10.1155/2022/7696251

**Published:** 2022-08-22

**Authors:** Yeming Wang, Tengchen Feng, Shutie Li, Ning Li, Zhanlong Yang, Xiaojia Sun, Fulong Li

**Affiliations:** ^1^Department of Anesthesiology, The First Affiliated Hospital of Hebei North University, Zhangjiakou, Hebei 075000, China; ^2^Department of Geriatrics, The First Affiliated Hospital of Hebei North University, Zhangjiakou, Hebei 075000, China; ^3^Operating Room, The First Affiliated Hospital of Hebei North University, Zhangjiakou, Hebei 075000, China

## Abstract

Angioneurotic headache is a common headache type in clinical treatment. At present, patients with nervous headache are mainly treated with oral western medicine in clinic, but it is usually difficult to obtain the ideal effect. In this study, we analyzed the effects of continuous lidocaine infusion through an ultrasound-guided cervical sympathetic ganglia (SG) catheter on cerebral hemodynamics and thermal imaging characteristics of head and neck in patients with angioneurotic headache and explored the clinical feasibility of this scheme. The results show that continuous infusion of lidocaine under ultrasound-guided SG catheterization can alleviate headache in patients with angioneurotic headache, which may be related to improving cerebral hemodynamics.

## 1. Introduction

Angioneurotic headache is one of the clinical chronic headache diseases, which can occur at all ages, especially in young and middle ages. It may be related to neurological disorders caused by great mental stress. Spasmodic constriction of the blood vessels in the head induces headache [1, 2]. The types of drugs clinically used for angioneurotic headaches include calcium ion antagonists, beta-blockers, antihistamines, antidepressants, and so on. Although the clinical treatment of headache symptoms is more effective, it cannot be cured and can only relieve headache symptoms. After stopping the drug, the headache symptoms will recur again, aggravating the pain of the patient's headache, inducing the negative emotions, and aggravating the psychological pressure of the patient. Repeated headache will form a vicious circle, affecting the patient's work and life [3–5]. The cervical sympathetic ganglion (SG) is the cervical ganglion composed of the sixth and seventh cervical nerves fused with the first thoracic ganglion to form the inferior cervical ganglion [6]. With the deepening of research on angioneurotic headache, medical workers have found that cervical sympathetic ganglia block (SGB) can inject local anesthetics into the loose connective tissue containing SG, so that the SGB nerves are innervated, thus effectively treating headache [7]. However, complications such as nerve injury and pneumothorax in conventional SGB are high in risk and are easily affected by insufficient puncture experience. However, the cervical sympathetic nerve block technique under the guidance of ultrasound can significantly improve the success rate and reduce the adverse reactions during the puncture. However, there are few reports regarding the treatment of angioneurotic headache with ultrasound-guided cervical sympathetic nerve block. This study explored the effects of continuous infusion of lidocaine through SG catheter under the guidance of ultrasound on cerebral hemodynamics and thermal imaging characteristics of head and neck in patients with angioneurotic headache.

## 2. Materials and Methods

### 2.1. General Information

80 patients with angioneurotic headache admitted to the hospital from May 2021 to May 2022 were selected and divided into the control group and the observation group by random number table, with 40 cases in each group. The subjects included in this study were informed about the study, voluntarily participated in the study, and signed the informed consent form, which was approved by the hospital ethics committee.

### 2.2. Inclusion Criteria

Inclusion criteria were as follows: meet the diagnostic criteria for angioneurotic headache [8]; patients who meet SGB indications [9]; and patients with good compliance during treatment.

### 2.3. Exclusion Criteria

Exclusion criteria were as follows: craniocerebral injury, traumatic brain injury, intracranial space-occupying lesions, cerebral infarction, and cerebral hemorrhage; nasal or drug-induced trigeminal headache; abnormal liver and kidney function, cardiac insufficiency, and coagulation dysfunction; headache due to liver and lung diseases; allergic to the drug used in the study; pregnancy and lactation; and hypertension and diabetes.

### 2.4. Methods

#### 2.4.1. Collection of Basic Patient Data

Through the hospital electronic case management system, the basic information of the patient is retrieved and entered in double copies. Basic information includes age, gender, course of disease, place of residence, drinking history, smoking history, headache location, and so on.

#### 2.4.2. Treatment Methods

The control group received traditional SGB treatment. The root of the anterior nodule of C6 transverse process, 1.5 cm away from the midline, and 2.5-3 cm cephalad of the sternoclavicular joint were used as the needle insertion points, and a 10 mL syringe was inserted perpendicular to the coronal plane to the root of the C6 transverse process. The depth of needle insertion is 1.5–3.5 cm. After no blood, spinal fluid, or gas is recovered, a mixed solution of 1% lidocaine [National Medicine Zhunzi H13022313, Hebei Tiancheng Pharmaceutical Co., Ltd.] and normal saline (5 mL 1% lidocaine + 5 mL of normal saline) was injected once a day, alternately on both sides, for 10 days of continuous treatment. The observation group was treated with continuous pumping of lidocaine with SG catheter under the guidance of ultrasound. The patient was placed in a supine position with the occiput removed, and the head was slightly tilted back. The ultrasound showed the transverse processes of C6 and C7, and the posterior edge of the sternocleidomastoid muscle was selected. Lateral approach, pay attention to avoid the thyroid, esophagus, blood vessels and nerves, and place a tube on the surface of the longus neck muscle at the level of the C7 transverse process. The lidocaine solution was 1 mL/h, the volume of each self-controlled pump was 1 mL, the locking time was 0.5 h, and the limit volume was 3 mL/h. The two operating physicians were the same person.

### 2.5. Observation Indicators and Detection Methods

#### 2.5.1. Record Indicators

The postoperative adverse reactions of the patients were recorded, including the number of headaches, the degree of headache, and the duration of each headache at 1 month (T1), 3 months (T3), and 6 months (T6) after surgery. Cerebral hemodynamics and head and neck thermal imaging changes were recorded.

#### 2.5.2. Numerical Rating Scale (NRS)

The scoring method can finely divide pain into 10 grades. The more severe the pain, the higher the score, which is no pain (0 points), mild pain (1–3 points), moderate pain (4–6 points), and severe pain (7–10 points).

#### 2.5.3. Detection of Cerebral Hemodynamic Indexes

Transcranial Doppler (TCD) was used to detect the changes of cerebral hemodynamics in patients. The parameters recorded were middle cerebral artery (MCA), anterior cerebral artery (ACA), posterior inferior cerebellar artery (PICA), vertebral artery (VA), and basilar artery (BA) blood flow.

#### 2.5.4. Infrared Thermal Imaging (IR-TI) Technology

To observe the thermal imaging changes of the patient's head and neck, the patient exposed the head and neck and waited for 20 minutes in a quiet state in the room. The DW-910 medical far-infrared thermal imager was used, and the focal length was set to 1.5∼2.0 m; the thermal image of the patient was collected, and IIRA special software was used to locate and quantitatively analyze the change of color code temperature value.

### 2.6. Statistical Method

SPSS 19.0 software was used for statistical analysis in this study, measurement data were expressed as mean ± standard deviation, *t*-test was used between groups, and repeated-measures analysis of variance was used for analysis of different time periods in the same group. The enumeration data were expressed as the number of cases (percentage), and the *χ*^2^ test was used for the analysis between groups (*a* = 0.05).

## 3. Results

### 3.1. Comparison of the Basic Data of the Two Groups of Patients

There was no statistical difference in the basic data of the two groups of patients (*P* > 0.05, Table 1).

### 3.2. Comparison of Postoperative Adverse Reactions and Headaches in the Two Groups of Patients

There was no statistical difference in postoperative blurred vision, decreased appetite, nausea and vomiting, rash, stomach pain, and postoperative adverse reactions between the two groups (*P* > 0.05, Table 2).

### 3.3. Comparison of Postoperative Headache in Two Groups of Patients

Compared with before operation, the number of headaches, NRS, and duration of each headache at time points T1, T3, and T6 in the two groups were decreased after operation (*P* < 0.05). At T1, T3, and T6 time points, the number of headaches, NRS, and duration of each headache in the observation group were lower than those in the control group (*P* < 0.05, Figure 1).

### 3.4. Comparison of Postoperative Cerebral Hemodynamics and Thermal Imaging Changes of Head and Neck between Two Groups of Patients

Compared with preoperative, MCA, ACA, PICA, VA, and BA at T1, T3, and T6 time points in the two groups were decreased (*P* < 0.05). At T1, T3, and T6 time points, the MCA, ACA, PICA, VA, and BA of the observation group were lower than those of the control group (*P* < 0.05). Compared with preoperative, the average color code temperature values of head and neck at T1, T3, and T6 time points in both groups were decreased (*P* < 0.05, Figure 2).

## 4. Discussion

The pathological mechanism of angioneurotic headache has not been clearly elucidated. There are currently vasoconstriction theory and self-limited neuritis theory on the pathogenesis of this disease. Emotional stress, mental stimulation, endocrine disorders, metabolic disorders, neuromodulation disorders, and sleep disorders are also the main causes of the disease. During the onset of the disease, one or both sides of the head may have recurring fluctuating pain. Some patients may also experience symptoms such as vomiting and nausea, which seriously affect the patients' daily life and works [10]. SG belongs to the cervical sympathetic ganglion, and the sympathetic nerve fibers from the SG can participate in the activities of the heart and blood vessels [11]. Studies have shown that SGB treatment can effectively reduce the severity of posttraumatic stress disorder and can be used as adjunctive treatments for posttraumatic stress disorder [12]. At the same time, SGB can also be used for the treatment of vascular neuropathic headache. It can relieve the excessive tension and hyperfunction of the ganglion and is conducive to the expansion of blood vessels in the head, neck, upper limbs, and heart. Thereby, it can improve blood flow, regulate the function of the endocrine system, and achieve the function of stabilizing the autonomic nerve function of the whole body [13, 14].

Although traditional SGB has achieved good results in the treatment of pain, it also has some drawbacks, for example, the operation is obviously empirical and the treatment effect is greatly affected by the operator himself [15]. In order to improve the safety of treatment, the process of using SG intubation and pumping anesthetic drugs under the real-time guidance of ultrasound not only accurately guides and locates the patient's drug delivery site but also avoids vascular damage and nerve damage during the puncture process and avoids the occurrence of intravascular drug injection accidents [16]. In addition, the continuous administration of analgesia pump can continuously deliver drugs around the nerves, and at the same time, it can control the dosage of drugs and realize personalized medicine. The results of this study showed that the number of headaches, NRS, and duration of each headache in the two groups at different times after treatment were significantly lower than those before surgery, and the decrease trend of the above indicators in the observation group was more obvious at the same time point after surgery [17]. This indicates that SGB treatment can improve the severity of headache in patients with angioneurotic headache, and the treatment effect of ultrasound-guided SG catheter with continuous infusion of lidocaine is more significant. Secondary vasoconstriction of intracranial arteries during headache attacks affects cerebral hemodynamics [18]. Thermal imaging is the result of infrared radiation through the thermal motion of molecules inside an object. It converts infrared energy into electrical signals and displays images and temperature values on the display. Local hyperthermia on thermal imaging suggests possible vascular disease [19, 20]. Observing the thermal imaging characteristics of head and neck in patients with angioneurotic headache before and after treatment is helpful to judge the changes of local cerebral blood perfusion and objectively and quantitatively analyze the treatment effect. This study also found that the cerebral hemodynamic indexes and the average color code temperature value of thermal imaging in the two groups of patients after treatment showed a significant decrease trend, indicating that SGB technology can significantly improve the cerebral blood flow in patients with angioneurotic headache.

Lidocaine is a class IB antiarrhythmic drug, which can block sodium ion channels and play a role in stabilizing the membrane. It is also an amide local anesthetic, and its anesthetic effect is twice that of procaine. Excessive drug doses can induce adverse reactions such as respiratory depression [21]. Lidocaine has been included in our country's Essential Drug List and can also be provided in primary hospitals. Therefore, in this study, the concentration of lidocaine continuously pumped by ultrasound-guided SG catheter was chosen to be 0.2% [22]. The results of this study showed that there was no statistical difference in the incidence of adverse events in patients with continuous pumping of lidocaine under ultrasound-guided SG catheterization compared with the incidence of adverse events in patients treated with conventional SGB. The concentration of the drug is lower than that used in conventional treatment, and the incidence of adverse reactions should be significantly reduced. However, the results of this study did not show such a trend, which may be related to the small number of cases included in this study, resulting in statistical analysis that cannot be presented. It is also possible that the conventional SGB treatment concentration is already an appropriate concentration with a therapeutic effect, so this study cannot observe significant differences by reducing the drug concentration again.

In conclusion, continuous pumping of lidocaine with SG catheter under ultrasound guidance can significantly reduce the severity and duration of headache in patients with angioneurotic headache and can also improve cerebral hemodynamics in patients with angioneurotic headache. However, this study still has a small number of cases and lacks multi-center exploration.

## Figures and Tables

**Figure 1:** Comparison of postoperative headache in two groups of patients. (a) The number of headaches. (b) NRS score. (c) The duration of each headache. Compared with the control group, ^*a*^*P* < 0.05; compared with preoperative, ^*b*^*P* < 0.05; compared with T1, ^*c*^*P* < 0.05; compared with T3, ^*d*^*P* < 0.05.

**Figure 2:** Comparison of postoperative cerebral hemodynamics and thermal imaging changes of head and neck between two groups of patients. (a) The number of headaches. (b) NRS score. (c) The duration of each headache. Compared with the control group, ^*a*^*P* < 0.05; compared with preoperative, ^*b*^*P* < 0.05; compared with T1, ^*c*^*P* < 0.05; compared with T3, ^*d*^*P* < 0.05.

**Table 1:** Comparison of the basic data of the two groups of patients.

Indexes	Control group (*n* = 40)	Observation group (*n* = 40)	*t*/*χ*^2^ value	*P* value
Age (year)	47.52 ± 5.26	47.85 ± 4.63	0.293	0.770
Gender			0.450	0.502
Male	21 (52.50)	18 (45.00)		
Female	19 (47.50)	22 (55.00)		
Course of disease (year)	3.20 ± 0.56	3.18 ± 0.59	0.193	0.847
Place of residence			0.238	0.626
Urban	29 (72.50)	27 (67.50)		
Rural	11 (27.50)	13 (32.50)		
Drinking history			0.051	0.822
Yes	23 (57.50)	22 (55.00)		
No	17 (42.50)	18 (45.00)		
Smoking history			0.220	0.639
Yes	27 (67.50)	25 (62.50)		
No	13 (32.50)	15 (37.50)		
Headache area			0.374	0.829
Left	14 (35.00)	12 (30.00)		
Right	24 (60.00)	25 (62.50)		
Bilateral	2 (5.00)	3 (7.50)		

**Table 2:** Comparison of postoperative complications and headache in two groups of patients.

Group	Control group (*n* = 40)	Observation group (*n* = 40)	*χ* ^2^ value	*P* value
Blurred vision	1 (2.50)	0 (0)	1.013	1.000
Decreased appetite	2 (5.00)	1 (2.50)	0.346	1.000
Feeling sick and vomiting	1 (2.50)	2 (5.00)	0.346	1.000
Rash	2 (5.00)	1 (2.50)	0.346	1.000
Stomach ache	2 (5.00)	1 (2.50)	0.346	1.000
Overall incidence	8 (20.00)	5 (12.50)	0.827	0.363

## Data Availability

The data used and/or analyzed during the current study are available from the corresponding author upon request.
